The article "Research on the Coordinated Development of New Rural Production and Living Civilization Construction from the Perspective of Green Transformation and Development" was published in 2022. Journal: Comput Intell Neurosci.

# Research on the Coordinated Development of New Rural Production and Living Civilization Construction from the Perspective of Green Transformation and Development

**DOI:** 10.1155/2022/1750256

**Published:** 2022-09-06

**Authors:** Xiaoyan Li

**Affiliations:** Xinyang Vocational and Technical College, Xinyang 464000, China

## Abstract

In order to improve the collaborative development effect of new rural production and living civilization construction, this article studies the collaborative development of rural production and living civilization construction combined with intelligent data processing algorithms and builds a model from the perspective of green transformation and development. In order to find as many and evenly distributed points as possible on the Pareto interface, a coevolution operator is designed in this article. The Pareto solutions of the two populations exchange information through the action of the co-occurrence operator and the absorption operator, so that the algorithm can find more and better noninferior solutions. The research shows that the collaborative development model of new rural production and living civilization construction has a certain effect, and it has a certain role in promoting the collaborative development of new rural production and living civilization construction.

## 1. Introduction

System civilization mainly includes economic system civilization and political system civilization. The so-called economic system refers to the economic basis at a certain stage of human history, that is, the sum of production relations [1]. Moreover, it is the foundation of political systems and social ideology. The economic system is the organization and operation mechanism of economic activities carried out by human beings to earn a living, and it is the concrete embodiment of the basic social economic system. Agriculture is the foundation of the development of the national economy, and the establishment of a distinctive socialist market economy system also includes the construction of the rural market economy system [2]. Since 80% of the population is in the countryside, this means that the productive force of the society is the rural productive force. Whether the economy can develop or not depends first on whether the rural areas can develop, and the key to rural development is the awakening of the self-awareness of rural productive forces. That is to say, the value embodiment of “institutional civilization” construction must first promote the healthy development of rural productive forces [3].

In the research on the value of ecological culture, Chen Shoupeng and Yang Lixin pointed out that the continuous development of society is due to the strong culture as the support and guarantee. As an advanced cultural form, ecological culture provides a strong driving force for the sustainable development of society. It is embodied in the fact that ecological culture provides the society with correct ecological values, ecological world outlook, ecological ethics, ecological science and technology, and ecological aesthetics, which is conducive to improving the civilization of the whole society [4]. Ecological culture is the key to solving the ecological crisis. It can not only provide ideological resources and theoretical references for improving human ecological awareness, but also promote the all-round development of human beings and the transition from modern production and lifestyle to ecological production and lifestyle [5]. While analyzing the value of ecological culture from the perspective of socialist culture construction, Lai Zhangsheng and Hu Xiaoyu believe that ecological culture should be an important part of characteristic socialist culture, which can enrich the new connotation of characteristic socialist harmonious culture and promote the innovation of characteristic socialist culture [6]. Ecological culture can lay a spiritual foundation for the construction of a socialist harmonious society, provide theoretical guidance for the concept of green development, and lay the groundwork for the construction of a socialist ecological civilization [7].

Rural ecological culture and ecological culture also have a narrow and broad difference. The broad rural ecological culture includes both the rural material production level and the ecological cultural content at the spiritual and institutional level; the narrow rural ecological culture specifically refers to the guidance of ecological values. The formed comprehensive cultural system, which covers rural “good” culture, awe culture, collectivism culture, and other cultural systems, not only pursues a friendly and harmonious system between man and nature, but also pursues the relationship between man and society [8]. From the perspective of the overall rural development, it is believed that rural ecological culture is a cultural form that coordinates various rural development and harmonious coexistence with nature, and the construction of rural ecological culture is one of the important means to ensure the harmonious, healthy, and sustainable development of rural areas in the ideological field [9]. For the problems existing in the development of rural ecological culture, due to the influence of traditional feudal concepts in rural areas, farmers' ecological awareness is weak, and their ecological cultural concepts are relatively backward. Moreover, the construction of rural ecological culture has just started; various systems and mechanisms are not perfect; and farmers pay too much attention to short-term interests, ignoring the long-term comprehensive social, economic, and ecological benefits of rural construction [10]. The problem of rural ecological culture construction is that the spiritual culture of farmers is insufficient; the brain drain is serious; and the support policies for ecological culture in rural areas are not perfect, lack guarantees, and have weak infrastructure [11]. From the perspective of spiritual, institutional, and material construction, the dilemma of rural ecological culture construction is manifested in the emptiness of farmers' ecological spiritual culture, the lack of ecological institutional culture, and the lack of ecological material culture [12].

The main way to build rural ecological culture is to change the current rural economic development mode, build an ecological agriculture industry system, continuously improve rural ecological facilities, and spread advanced culture and promote excellent traditional culture [13]. More detailed suggestions are made on the development of rural ecological culture. It is believed that the construction of rural ecological culture should shape and cultivate the traditional rural production and life style ecologically from the material form, and regulate and constrain the rural governments, social organizations, and enterprises at all levels from the institutional form. The majority of farmers spiritually establish the concept of ecological civilization of farmers [14]. The development of ecological culture requires an economic foundation. The construction of beautiful villages cannot be separated from the emerging economic foundation of rural areas. Second, the government should play a leading role and strengthen the protection of ecosystems [15]. In addition to promoting the transformation of rural economic development and enhancing the quality of farmers, Yang Rongrong believes that it is also necessary to build a good social environment and cultivate a strong social atmosphere. Some scholars have proposed to inherit and protect rural ecological culture and build ecological cultural reserves [16]. Scholars have made suggestions for the government, farmers, carrier construction, etc. The ultimate goal is to better develop rural ecological culture, completely change the unreasonable production and lifestyle in rural areas, and build a pattern of harmonious coexistence between rural people and nature [17].

Eco-Marxism mainly considers the causes of ecological crisis, the solution path, and the idea of ecological socialism. Ecological Marxism believes that the emergence of ecological crisis is due to the concept of human control of nature [18]. Ecological Marxism believes that the origin of ecological crisis lies in the capitalist system. Capitalism is a self-expanding system of economic development. Its purpose is the infinite growth of capital, while nature cannot expand infinitely. The contradiction between nature and capitalism is uncoordinated. Moreover, the ecological environment appears to be the alienation of the relationship between man and nature, but in fact it is the alienation of the practice subject under the capitalist system [19]. The best choice to protect the natural environment is to choose advanced socialism because socialism can overcome the contradiction between the expansion of capital profits and ecology, and realize the renewal of the entire mode of production. The thought of ecological Marxism seeks the insights of Marxism from the perspective of ecology, which has a positive enlightenment significance for the current handling of economic development and environmental protection [20].

This article studies the coordinated development of rural production and living civilization construction in combination with intelligent data processing algorithms, and constructs a model from the perspective of green transformation and development to provide a reference for the subsequent coordinated development of rural production and living civilization construction.

## 2. Intelligent Agriculture Development Data Analysis Algorithm

### 2.1. Basic Theory of Evolutionary Algorithms and Basic Concepts of Multiobjective Optimization

The principle of genetic algorithm is essentially based on Darwin's theory of natural selection. Usually, it is necessary to use a small selection pressure (to explore a certain breadth of the search space) in the early stage of genetic search, and use a large selection pressure (to limit the search space) in the late stage. The direction of the genetic search is directed to some of the more useful regions of the search space. The selection methods usually used are as follows: roulette wheel selection, (*μ*+*λ*) selection, tournament selection, elitist selection, and other forms.

Wheel selection method determines the selection probability of the individual according to the ratio of each chromosome fitness value. The probability of each individual entering the next generation is equal to the ratio of its fitness value to the sum of the fitness values of the individuals in the entire population. The higher the fitness value, the greater the probability of the individual being selected, and the greater the probability of the individual entering the next generation. The specific principle is as follows:

① The algorithm calculates the probability *P*_*i*_=Fit(*x*_*i*_)/∑_*j*=1_^*N*^Fit(*x*_*j*_),  *i*=1,2, ⋯, *N*, of the initial selection of each individual in the population, and the sum of the fitness of individuals in the population is ∑_*j*=1_^*N*^Fit(*x*_*j*_), where Fit(*x*_*j*_) is the fitness value of the individual *x*_*j*_.
② The algorithm calculates the cumulative probability *q*_*i*_=∑_*j*=1_^*i*^*P*_*j*_,  *i*=1,2, ⋯, *N* of each individual in the population.
③ The algorithm generates a random number *r* ∈ [0,1] according to a uniform distribution.
④ If *r* ≤ *q*_1_, the algorithm chooses *x*_1_; otherwise, if *q*_*i*_ < *r* ≤ *q*_*i*+1_, 1 ≤ *i* < *N* − 1, the algorithm chooses *x*_*i*+1_. If *k* < *N*, the algorithm sets *k*=*k*+1 and turns to ③; otherwise, the algorithm stops.

As shown in Figure 1, *q*_1_=*p*_1_=0.45, *q*_2_=*P*_1_+*P*_2_=0.75, *q*_3_=*P*_1_+*P*_2_+*P*_3_=0.95, *q*_4_=*P*_1_+*P*_2_+*P*_3_+*P*_4_=1, *x*_1_ has the highest probability of being selected into the next generation, and *x*_4_ has the lowest probability of being selected into the next generation.

The algorithm assumes that two individuals *x*_*i*_^*t*^ and *x*_*j*_^*t*^ are arithmetically crossed, and the two new individuals generated after the crossover are as follows:

(1) $$\begin{array}{c} \left\{\begin{array}{c} x_{i}^{t+1}=\alpha x_{j}^{t}+\left(1-\alpha \right)x_{i}^{t},\\ x_{j}^{t+1}=\alpha x_{i}^{t}+\left(1-\alpha \right)x_{j}^{t}. \end{array}\right. \end{array}$$

Among them, *α* ∈ [0,1] is a random number. In the main operation process of arithmetic crossover, ① the algorithm randomly generates the coefficient a when two individuals are linearly combined; ② the algorithm generates two new individuals according to formula (1).

#### 2.1.1. Mutation Operator

The genetic algorithm solves problems with the help of the principles and ideas of biological evolution. The following is the basic flow chart of genetic algorithm (Figure 2):

The following multiobjective problem is considered.

(2) $$\begin{array}{c} \min\underset{x\in \Omega }{F\left(x\right)}=\left(f_{1}\left(x\right),f_{2}\left(x\right),\cdots ,f_{M}\left(x\right)\right). \end{array}$$

Among them, *x*=(*x*_1_, *x*_2_, ⋯, *x*_*n*_) is an *n*-dimensional vector, Ω is the feasible solution space, and *f*_1_(*x*), *f*_2_(*x*), ⋯, *f*_*M*_(*x*) is *m-*objective functions. Generally, for a single-objective optimization problem, the global optimal solution is the solution that makes the objective function optimal. However, for a multiobjective optimization problem such as formula (2), usually, the functions to be optimized of *f*_1_(*x*), *f*_2_(*x*), ⋯, *f*_*M*_(*x*) are in conflict with each other, and they cannot achieve the desired optimal value at the same time. Scholars thought of using Pareto optimal solution to describe the solution of this optimization problem, in which multiple objective functions have conflicting functions. Pareto optimal solution is a commonly used definition of multiobjective optimization. The following basic definitions are now given:

**Definition 1 .**

A vector *u*=(*u*_1_, *u*_2_, ⋯, *u*_*M*_) is said to be noninferior to another vector *v*=(*v*_1_, *v*_2_, ⋯, *v*_*M*_), if and only if ∀*i* ∈ {1,2, ⋯, *M*} has *u*_*i*_ ≤ *v*_*i*_ and ∃*j* ∈ {1,2, ⋯, *M*} to makes *u*_*j*_ < *v*_*j*_.

**Definition 2 .**

In the Pareto optimal solution, for any two points *x*_1_, *x*_2_ ∈ Ω, if the following conditions hold:

(3) $$\begin{array}{c} \left\{\begin{array}{c} f_{i}\left(x_{1}\right)\leq f_{i}\left(x_{2}\right),\forall i\in \left\{1,2,\cdots ,M\right\},\\ f_{j}\left(x_{1}\right)<f_{j}\left(x_{2}\right),\exists j\in \left\{1,2,\cdots ,M\right\}. \end{array}\right. \end{array}$$

If vector (*f*_1_(*x*_1_), *f*_2_(*x*_1_), ⋯, *f*_*M*_(*x*_1_)) is better than vector (*f*_1_(*x*_2_), *f*_2_(*x*_2_), ⋯, *f*_*M*_(*x*_2_)), then *x*_1_ is said to be better than *x*_2_. It can be seen from the first condition of formula (3) that for *M* targets, *x*_1_ is no worse than *x*_2_. It can be seen from the second condition that *x*_1_ is better than *x*_2_ in at least one objective. Therefore, *x*_1_ should indeed be better than *x*_2_ when formula (3) is satisfied.

**Definition 3 .**

If there is no better solution than *x*_1_, in Ω, then *x*_1_, is said to be a Pareto optimal solution (or an efficient solution, or a noninferior solution) of formula. (2).

**Definition 4 .**

In the Pareto optimal solution set, for formula (2), the set *E*(*f*, Ω)={*x* ∈ Ω*|x* is called the Pareto optimal solution (or effective solution set or noninferior solution set) of formula (2).

**Definition 5 .**

In the Pareto frontier, for formula (2), the set

(4) $$\begin{array}{c} FE\left(f,\Omega \right)=\left\{\left(f_{1}\left(x\right),f_{2}\left(x\right),\cdots ,f_{M}\left(x\right)\right)|x\in E\left(f,\Omega \right)\right\}, \end{array}$$

is called the Pareto frontier (or effective frontier) of formula (2).

Figure 3 shows the Pareto optimal solution set and the corresponding Pareto front for a problem with two-objective functions as independent variables.

Ω is the decision variable space, where

(5) $$\begin{array}{c} Y=\left\{y\in R^{M}|y=\left(f_{1}\left(x\right),f_{2}\left(x\right),\cdots ,f_{M}\left(x\right)\right),x\in \Omega \right\}, \end{array}$$

is the objective function space.

The optimal solution of a multiobjective optimization problem is always on the boundary line (or surface) of the search area. As shown in Figure 4, the thick line segment represents the optimal interface (Pareto frontier) of the two-objective optimization. The optimal interface of three-objective optimization is a surface, and the optimal interface of three or more objectives constitutes a hypersurface. The solid points *A*, *B*, *C*, *D*, and *E* in Figure 4 are all on the optimal boundary, and they are all Pareto solutions, and they are nondominated with each other. However, the hollow points *F*, *G*, *H*, *I*, and *J* are not on the optimal boundary within the search area, so they are not optimal solutions, but dominated. Moreover, it is directly or indirectly governed by the optimal solution above the optimal boundary.

The commonly used methods for solving multiobjective optimization problems are as follows: weighted sum method, constraint method, objective programming method, max-min method, and so on.

*(1) Weighted Sum Method*. The weighted sum method can be expressed as follows: for each subobjective function *f*_*i*_(*x*), (*i*=1,2, ⋯, *M*), a different weight *ω*_*i*_ ≥ 0(*i*=1,2, ⋯, *M*) is assigned as the coefficient of each objective function, and ∑_*i*=1_^*M*^*ω*_*i*_=1. The linear weighted sum of each subobjective function is expressed as follows:

(6) $$\begin{array}{c} \left\{\begin{array}{cc} \min & f\left(x\right)=\sum_{i=1}^{M}\omega_{i}f_{i}\left(x\right),\\ \text{s.t}. & x\in \Omega . \end{array}\right. \end{array}$$

Thousands of different Pareto optimal solutions are obtained by choosing thousands of different weight combinations. This method is extremely simple, but it is also a more classical method for solving multiobjective optimization problems. Its advantage is that it is well understood and easy to calculate; its disadvantage is that the selection of weights is related to the relative importance of each target. In addition, the weighted sum method is sensitive to the shape of the Pareto interface, and the optimal solution for the convex part of the Pareto interface cannot be obtained.

*(2) *ε*-Constrained Method*. The main idea of this method is to use the important objective function of multiobjective optimization as the optimization objective, while other objective functions are used as constraint functions to solve. The optimization problem transformed by this constraint method is expressed as follows:

(7) $$\begin{array}{c} P_{k}\left(\varepsilon_{k}\right)\left\{\begin{array}{c} \min f_{k}\left(x\right),\\ s.t.f_{j}\left(x\right)\leq \varepsilon_{j}^{k},x\in \Omega ,1,1\leq j\leq k. \end{array}\right. \end{array}$$

The advantage of this method is that it is easy to operate, where different values of *ε*_*j*_ are selected during the optimization process, and multiple Pareto optimal solutions can be found, which is very practical in practical problems. However, the disadvantage is that certain prior knowledge is usually required to select a suitable *ε*_*j*_, and this prior knowledge is usually unknown.

There are many types of multiobjective evolutionary algorithms (MOE), and the methods they use are also very different, which is difficult to describe by a general framework. For the convenience of understanding, we design a flowchart of a multiobjective evolutionary algorithm based on Pareto optimality (Figure 5).

It assumes that there are *n* factors, each with *q* levels. When *n* and *q* are given, the purpose of uniform design is to find *q* combinations from all *q*^*n*^ combinations so that the *q* combinations are uniformly distributed in all possible combination spaces.

(8) $$\begin{array}{c} U\left(n,q\right)={\left[U_{i,j}\right]}_{q\times n}. \end{array}$$

It means that the selected *q* combinations are uniformly distributed, where *U*_*i*,*j*_ represents the level of the *j*-th factor in the *i*-th combination. When *q* is prime and *q* > *n*, it has been shown that *U*_*i*,*j*_ can be calculated as follows:

(9) $$\begin{array}{c} U_{i,j}=\left(i\sigma^{j-1}\mathrm{mod}q\right)+1. \end{array}$$

The values of *σ* are listed in Table 1.

### 2.2. A Multiobjective Coevolutionary Algorithm Based on Uniform Design

In multiobjective optimization, each objective function value has different orders of magnitude. If only the simple weighted summation of the objective function is used as the fitness function, then the value of the fitness function will be dominated by the one with the larger order of magnitude of the objective function value. For example, for two-objective optimization, *f*_1_(*x*) represents cost, and its value range is 300 ≤ *f*_1_(*x*) ≤ 500, *f*_2_(*x*) represents reliability, and its value range is 0 ≤ *f*_2_(*x*) ≤ 1. Then, the value of *ω*_1_*f*_1_(*x*)+*ω*_2_*f*_2_(*x*) will be dominated by *f*_1_(*x*). To avoid similar situations, we normalize the objective function as follows:

(10) $$\begin{array}{c} h_{i}\left(x\right)=\frac{f_{1}\left(x\right)}{\max_{y\in \Omega }\left\{\left|f_{1}\left(y\right)\right|\right\}}. \end{array}$$

Among them, Ω is the point set of the current population, and *h*_*i*_(*x*) is the normalized objective function.

For a given *N*, the constructed *N* fitness functions are as follows:

(11) $$\begin{array}{c} {\text{fitness}}_{i}=\omega_{i,1}h_{1}\left(x\right)+\omega_{i,2}h_{2}\left(x\right)+\cdots +\omega_{i,M}h_{M}\left(x\right),1\leq i\leq N. \end{array}$$

Among them, *ω*_*i*_=(*ω*_*i*,1_, *ω*_*i*,2_, ⋯, *ω*_*i*,*M*_) is the weight vector, and *ω*_*i*,*j*_ ≥ 0, *j*=1,2, ⋯, *M*, ∑_*j*=1_^*M*^*ω*_*i*,*j*_=1.

In order to make the search approach to the Pareto front evenly, a uniform design method is used to construct the weight vector. In the target space, considering each target as a factor, there are *M* factors to construct *N* fitness functions, then *N* weight vectors are needed, and each factor takes *N* levels. Then, using the uniform array *U*(*M*, *N*), *ω*_*i*,*j*_(*i*=1,2, ⋯, *N*; *j*=1,2, ⋯, *M*) is calculated as follows:

(12) $$\begin{array}{c} \omega_{i,j}=\frac{U_{i,j}}{U_{i,1}+U_{i,2}+\cdots +U_{i,M}}. \end{array}$$

**Example 1 .**

The *M*=3, *q*=5 means that there are 3 objective functions, and 5 uniformly distributed weight vectors are to be generated, that is, a uniform array with 3 factors and 5 levels is constructed. It can be seen from Table 1 that *σ*=2, and the uniform array is generated by formula (6)

Then, according to formula (3), 5 weight vectors are generated, and then formula (3) is used to construct the corresponding fitness function:

*l*=(*l*_1_, *l*_2_, ⋯, *l*_*N*_), *u*=(*u*_1_, *u*_2_, ⋯, *u*_*N*_) Among them, [*l*, *u*] is the feasible region, if *x*=(*x*_1_, *x*_2_, ⋯, *x*_*N*_) ∈ [*l*, *u*], *x* is called a feasible solution of the problem. [*l*, *u*] is divided into *H* different subspaces [*l*(1), *u*(1)], [*l*(2), *u*(2)],…, [*l*(*H*), *u*(*H*)], and the parameter H can take the value 2, 2^2^, or 2^3^ and so on.

The solution interval is divided into two subspaces in the following manner. First, the component with the largest value range is selected, then the solution space is equally divided into two subspaces along the direction of this component, and then the two subspaces are divided into four subspaces according to this method. For any subspace, such as [*l*(1), *u*(1)], the coordinate axis with the largest value range is selected, and the two subspaces are divided into four subspaces along this coordinate direction. The above process is repeated until the solution space is divided into H subspaces. The following is the specific algorithm.

Among them, *k*=(*j*_1_ − 1)*n*_2_*n*_3_ ⋯ *n*_*N*_+(*j*_2_ − 1)*n*_3_*n*_4_ ⋯ *n*_*N*_+⋯+(*j*_*N*_ − 1)*n*_*N*_+*j*_*N*_.

After the algorithm divides the solution space into *H* subspaces, the sample points are selected for each subspace according to the following methods. The algorithm considers an arbitrary subspace, such as the *k*-th subspace, and denotes it as follows:

(13) $$\begin{array}{c} \left[l\left(k\right),u\left(k\right)\right]=\left[\left(l_{1}\left(k\right),l_{2}\left(k\right),\cdots ,l_{N}\left(k\right)\right),\left(u_{1}\left(k\right),u_{2}\left(k\right),\cdots ,u_{N}\left(k\right)\right)\right]. \end{array}$$

In this subspace, the algorithm discretizes the value range of *x*_*i*_ into *Q* levels *α*_*i*,1_(*k*), *α*_*i*,2_(*k*), ⋯, *α*_*i*,*Q*_(*k*), where *Q* is a parameter and is a prime number, and *a*_*i*,*j*_(*k*) is calculated according to the following formula:

(14) $$\begin{array}{c} a_{i,j}\left(k\right)=\left\{\begin{array}{cc} l_{1}\left(k\right), & j=1,\\ l_{1}\left(k\right)+\left(j-1\right)\frac{u_{i}\left(k\right)-l_{i}\left(k\right)}{Q-1}, & 2\leq j\leq Q-1,\\ u_{1}\left(k\right), & j=Q. \end{array}\right. \end{array}$$

According to Algorithm 1, it can be known that the difference between any two adjacent levels is the same. It is recorded as *α*_*i*_(*k*)=(*α*_*i*,1_(*k*), *α*_*i*,2_(*k*), ⋯, *α*_*i*,*Q*_(*k*)), after discretizing the value area of *x*_*i*_ into *Q* levels, there will be *Q*^*N*^ points in each subspace. Then, a uniform array *U*(*N*, *Q*) is used to select *Q* sample points in each subspace, denoted as follows:

(15) $$\begin{array}{c} \left\{\begin{array}{c} \left(\alpha_{1,U_{1,1}}\left(k\right),\alpha_{2,U_{1,2}}\left(k\right),\cdots ,\alpha_{N,U_{1,N}}\left(k\right)\right),\\ \left(\alpha_{1,U_{2,1}}\left(k\right),\alpha_{2,U_{2,2}}\left(k\right),\cdots ,\alpha_{N,U_{2,N}}\left(k\right)\right),\\ \cdots \\ \left(\alpha_{1,U_{Q,1}}\left(k\right),\alpha_{2,U_{Q,2}}\left(k\right),\cdots ,\alpha_{N,U_{Q,N}}\left(k\right)\right). \end{array}\right. \end{array}$$

The algorithm performs the above operations on all *H* subspaces, with a total of *HQ* sample points.

Among the *HQ* sample points, pop points are selected as the initial population. To search in *D* directions, *D* fitness functions are constructed, where *D* is a parameter and a prime number. Through each fitness function, all *HQ* points are evaluated to select the best ⌊pop/*D*⌋, and finally a total of pop points are selected to form an initial group. The specific algorithm is as follows.

**Example 2 .**

The algorithm considers a two-dimensional solution space: the algorithm sets 1 ≤ *x*_1_ ≤ 4, −20 ≤ *x*_2_ ≤ 10 and its feasible solution area [*l*, *u*] is [(1, −20)(4,10)]. The parameters are set as follows: *H*=4, *Q*=5, *D*=6, *pop*=10. Algorithm 1 is executed to divide the solution space into the following four subspaces, and Algorithm 2 is executed to generate the initial population:

(1) According to Algorithm 1, there are *a*=(1, −20), *z*=(4,10).
(2) Among them, Δ_1_=3, Δ_2_=7.5, *n*_1_=1, *n*_2_=4, and the following four subspaces are obtained after division:
  (16) $$\begin{array}{c} \left\{\begin{array}{c} \left[l\left(1\right),u\left(1\right)\right]=\left[\left(1,20\right),\left(4,-12.5\right)\right],\\ \left[l\left(2\right),u\left(2\right)\right]=\left[\left(1,-12.5\right),\left(4,-5\right)\right],\\ \left[l\left(3\right),u\left(3\right)\right]=\left[\left(1,-5\right),\left(4,23,.5\right)\right],\\ \left[l\left(4\right),u\left(4\right)\right]=\left[\left(1,20\right),\left(4,-12.5\right)\right]. \end{array}\right. \end{array}$$
Next, Algorithm 2 is performed to generate the initial population.
(3) The result obtained by discretizing the first subspace [*l*(1), *u*(1)]=[(1,20), (4, −12.5)] according to formula (11) is as follows:
  (17) $$\begin{array}{c} \left\{\begin{array}{c} \alpha_{1}\left(1\right)=\left(1,1.75,2.5,3,25,4\right),\\ \alpha_{2}\left(1\right)=\left(-20,-10.125,-16-23,-14,375,-12.5\right). \end{array}\right. \end{array}$$
Then, according to the uniform array $U=\left(2,5\right)=\left[\begin{array}{ccccc} 2 & 3 & 4 & 5 & 1\\ 3 & 5 & 2 & 4 & 1 \end{array}\right]$ and formula (3), five sample points are selected as follows:
  (18) $$\begin{array}{c} \left\{\begin{array}{c} \left(1.75,-16.5\right),\\ \left(2.5,-12.5\right),\\ \left(3.25,-18.125\right),\\ \left(4,-14.375\right),\\ \left(1,-20\right). \end{array}\right. \end{array}$$
The algorithm performs similar operations on the other three subspaces, and a total of 20 sample points are obtained.
(4) The algorithm evaluates the 20 sample points according to the five fitness functions, each fitness function selects [20/10]=2 best points, and a total of 10 sample points are selected from the five fitness functions to form the initial group.

### 2.3. Genetic Operator

Symbiotic operators *P*_*t*_^*a*^=(*P*_1_^*a*^, *P*_2_^*a*^, ⋯, *P*_*M*_^*a*^) and *P*_*t*_^*b*^=(*P*_1_^*b*^, *P*_2_^*b*^, ⋯, *P*_*M*_^*b*^) are two parent groups, and the corresponding nondominated solution sets are denoted as *O*_*t*_^*a*^ and *O*_*t*_^*b*^, respectively. For any (*x*_1_^*a*^, *x*_2_^*a*^, ⋯, *x*_*n*_^*a*^) in the population *P*_*t*_^*a*^, an individual (*o*_1_^*b*^, *o*_2_^*b*^,…, *o*_*n*_^*b*^) is randomly selected in *O*_*t*_^*b*^. Afterwards, a new individual is generated according to the following formula, denoted as (*z*_1_^*a*^, *z*_2_^*a*^, ⋯, *z*_*n*_^*a*^), and the next generation group product is generated. Among them, *r* represents a uniform number randomly distributed in [−1,1].

(19) $$\begin{array}{c} z_{i}^{a}=o_{i}^{b}+r\cdot \left(o_{i}^{b}-x_{i}^{a}\right),\;i=1,2,\ldots ,n. \end{array}$$

In the same way, for any individual (*x*_1_^*b*^, *x*_2_^*b*^,…, *x*_*n*_^*b*^) in the group *P*_*t*_^*b*^, the algorithm randomly selects an individual (*o*_1_^*a*^, *o*_2_^*a*^,…, *o*_*n*_^*a*^) in *O*_*t*_^*a*^ and generates a new individual (*z*_1_^*b*^, *z*_2_^*b*^,…, *z*_*n*_^*b*^) according to the following formula, and then, the next generation of group *p*_*t*+1_^*a*^ is generated.

(20) $$\begin{array}{c} z_{i}^{b}=o_{i}^{a}+r\cdot \left(o_{i}^{a}-x_{i}^{b}\right),\;i=1,2,\ldots ,n. \end{array}$$

*P*_*t*_^*a*^ and *P*_*t*_^*b*^ are two groups that have evolved separately, that is, search in different spatial regions in the variable space. By the function of formulas (13) and (14), the two groups exchange information with each other.

Attraction operators *P*_*t*_^*a*^=(*X*_1_, *X*_2_,…, *X*_*M*_) and *P*_*t*_^*b*^=(*Y*_1_, *Y*_2_,…, *Y*_*M*_) are two parent groups, and the corresponding nondominated solution sets are denoted as *O*_*t*_^*a*^ and *O*_*t*_^*b*^, respectively. If

(21) $$\begin{array}{c} \forall X\in O_{t}^{a},\exists Y\in O_{t}^{b},Y>X, \end{array}$$

is established, then the group *P*_*t*_^*b*^ absorbs the group *P*_*t*_^*a*^ to generate a new group *P*_*t*+1_^*b*^(*l*_1_, *l*_2_,…, *l*_*N*+*M*_). Among them, *l*_*i*_=*Y*_*i*_, *i*=1,2,…, *N*, and *l*_*i*_, *i*=*N*+1, *N*+2,…, *N*+*M* is generated by:

(22) $$\begin{array}{c} l_{i,j}=o_{j}+r\cdot \left(o_{j}-x_{i-N,j}\right),\;j=1,2,\ldots ,n. \end{array}$$

From the above expression, we can know that *O*_*t*_^*b*^ is better than *O*_*t*_^*a*^, that is, the solution in group *P*_*t*_^*b*^ is better than the solution in group *P*_*t*_^*a*^. In this case, it is much less likely that the quality of the solution obtained by evolving population *P*_*t*_^*a*^ is better than the quality of the solution obtained by de-evolving population *P*_*t*_^*b*^. Therefore, in this competition, group *P*_*t*_^*a*^ will inevitably disappear. In addition, there may be some relatively useful information in the group *P*_*t*_^*a*^, which can be utilized by (16) to generate better or useful individuals.

Discrete operator: the population *P*_*t*_^*a*^=(*P*_1_^*a*^, *P*_2_^*a*^, ⋯, *P*_*M*_^*a*^) is randomly discretized into two subpopulations, denoted as *P*_*t*_^*ta*^=(*Z*_1_^*a*^, *Z*_2_^*a*^,…, *Z*_*M*/2_^*a*^) and *P*_*t*_^*tb*^=(*Z*_1_^*b*^, *Z*_2_^*b*^,…, *Z*_*M*/2_^*b*^), respectively. A population is randomly selected, and the algorithm takes *P*_*t*_^*ta*^ and performs the following mutation operations on each individual in *P*_*t*_^*tb*^:

(23) $$\begin{array}{c} z_{k}^{a}=\left\{\begin{array}{c} z_{k}^{a}+\frac{\left(u_{k}^{a}-l_{k}^{a}\right)}{t}\cdot rr\leq 0.5,\\ z_{k}^{a}-\frac{\left(u_{k}^{a}-l_{k}^{a}\right)}{t}\cdot \text{otherwise}, \end{array},\;k=1,2,\ldots ,n\right.. \end{array}$$

Among them, *r* represents the uniform number randomly distributed in the [0,1] interval, and *t* represents the evolutionary algebra. *u*_*k*_^*a*^ and *l*_*k*_^*a*^ are the upper and lower bounds of the k-th coordinate of the point in the search space, respectively. The purpose of doing this is that there may be some more useful information in the group *P*_*t*_^*a*^. After the group *P*_*t*_^*a*^ is acted on by a discrete operator, a new individual is obtained and the diversity of the group is increased. It is also possible to obtain some solutions that are better than the current population, or to find solutions for nonconvex parts of the Pareto interface.

## 3. Research on the Coordinated Development of New Rural Production and Living Civilization Construction from the Perspective of Green Transformation and Development

The energy system diagram reflects the basic structure inside each system and the relationship between energy and matter inside and outside the system. The level of the energy conversion rate of each legend and its respective components determine the arrangement order of the legends inside and outside the boundary of the system diagram, and the energy conversion rate decreases from right to left, as shown in Figure 6.

## 4. Simulation Test Research

This article proposes a method for calculating the degree of distribution, which is used to measure whether the Pareto optimal solution set obtained by the algorithm is uniformly distributed in the target space. The function is defined as follows:

(24) $$\begin{array}{c} S=\sqrt{\frac{1}{\left|Q\right|-1}\sum_{i=1}^{\left|Q\right|}{\left(d_{i}-\bar{d}\right)}^{2}}. \end{array}$$

Among them,

(25) $$\begin{array}{c} d_{1}=\underset{j\in Q\wedge j\neq 1}{\min}\sum_{k=1}^{m}\left|f_{k}^{i}-f_{k}^{j}\right|,\bar{d}=\left(\frac{\sum_{i=1}^{\left|Q\right|}d_{1}}{\left|Q\right|,i,j\in Q}\right), \end{array}$$

where *m* is the number of objective functions, and *Q* is the set of nondominated solutions obtained by the algorithm. |*Q*| represents the number of elements in the nondominated solution set “*Q*.” The value of *S* is the *S* metric. When the solutions in the set *Q* tend to be uniformly distributed, the smaller the value of the corresponding distance evaluation function *S* is, the more uniformly the noninferior solution set obtained by the algorithm is distributed in the target space.

The measure of broadness (maximum spread) mainly compares the performance of the algorithm by calculating the perimeter of the polyhedron formed by all extreme values in the solution set P, which is defined as follows:

(26) $$\begin{array}{c} M=\sqrt{\sum_{k=1}^{m}{\left(\max_{i}^{N}f_{k}^{i}-\min_{t}^{N}f_{k}^{l}\right)}^{2}}. \end{array}$$

Among them, *N* is the number of nondominated solutions, and *m* is the dimension of the target space. The larger the value of *M*, the wider the range of the solution set *P*, and the value of *M* is called the *M* measure.

To verify the effectiveness of the proposed new algorithm, the following test functions are selected.

(27) $$\begin{array}{c} \text{uestionone}\left\{\begin{array}{c} \min f_{1}\left(x\right)=\frac{1}{x_{1}^{2}+x_{2}^{2}+1},\\ \min f_{2}\left(x\right)=x_{1}^{2}+3x_{2}^{2},\\ \text{subject to}-3\leq x_{1}\leq 3,\\ -5\leq x_{2}\leq 5, \end{array}+1\right.\\ \text{questiontwo}\left\{\begin{array}{c} \min f_{1}\left(x\right)=2\sqrt{x_{1},}\\ \min f_{2}\left(x\right)=x_{1}\left(1-x_{2}\right)+5,\\ \text{subject to}1\leq x_{1}\leq 4,\\ 1\leq x_{2}\leq 2, \end{array}\right.\\ \text{questionthree}\left\{\begin{array}{c} \min f_{1}\left(x\right)=x_{1}^{2}+x_{2}^{2},\\ \min f_{2}\left(x\right)={\left(x_{1}-5\right)}^{2}+{\left(x_{2}-5\right)}^{2},\\ \text{subject to}-5\leq x_{1}\leq 10,\\ -5\leq x_{2}\leq 10, \end{array}\right.\\ \text{questionfour}\left\{\begin{array}{c} \min f_{1}\left(x\right)=1-\exp\left(-{\left(x_{1}-1\right)}^{2}-{\left(x_{2}+1\right)}^{2}\right),\\ \min f_{2}\left(x\right)=1-\exp\left(-{\left(x_{1}+1\right)}^{2}-{\left(x_{2}-1\right)}^{2}\right),\\ \text{subject to}-10\leq x_{1}\leq 10,\\ -10\leq x_{2}\leq 10. \end{array}\right. \end{array}$$

Figures 7to 10 visually compare the nondominated solution sets obtained by the algorithm UCEMOA in this article and the classical algorithm NSGA-II in a certain run.

It can be seen from Figures 6-8 that the algorithm UCEMOA obtains more noninferior solutions than NSGA-II. The following intervals are for the horizontal axis unless otherwise specified. It can be seen from 5 that between the interval [0, 0.1] and [0.6, 0.9], the algorithm UCEMOA in this article obtains more and uniformly distributed noninferior solutions than NSGA-II. It can be seen from Figure 6 that for the nonconvex Pareto optimal solution interface, the algorithm UCEMOA searches for more uniformly distributed and broad noninferior solutions than NSGA-II. It can be seen from Figure 7 that in the interval [0, 4], the algorithm UCEMOA in this article obtains more uniformly distributed and broad noninferior solutions than NSGA-II. In the interval [30, 50], our algorithm UCEMOA searches more noninferior solutions than NSGA-II. It can be seen from Figure 8 that in the interval [0, 0.5], the algorithm UCEMOA in this article obtains more noninferior solutions than NSGA-II. On the vertical axis, in the interval [0, 0.4], the algorithm UCEMOA in this article searches for more and uniformly distributed noninferior solutions than NSGA-II. Therefore, the algorithm UCEMOA can effectively search for the Pareto optimal solution, not only for the convex Pareto optimal solution interface problem, but also for the nonconvex Pareto optimal solution interface problem.

Based on the above analysis, the effect of the collaborative development model of new rural production and life civilization construction proposed in this article is evaluated, and the experimental results shown in Figure 11 are obtained.

It can be seen from the above research that the collaborative development model of new rural production and living civilization construction has a certain effect, and has a certain role in promoting the collaborative development of new rural production and living civilization construction.

## 5. Conclusion

Scientific research is always carried out under certain preconditions. The study of rural revitalization and the construction of rural civilization also has its own profound motivation. From the perspective of rural revitalization, the construction of rural-style civilization contains major theoretical problems faced by contemporary society, and the construction of rural-style civilization from the perspective of rural revitalization is a major academic issue worthy of in-depth study. Moreover, the construction of rural civilization from the perspective of rural revitalization is a major practical problem faced by contemporary society. In addition, the problem of rural development is a worldwide problem with universal significance. Therefore, being familiar with the research on the development of the country's rural society in foreign academic circles undoubtedly has important comparison and reference value for the writing of this article. This article studies the coordinated development of rural production and living civilization construction combined with intelligent data processing algorithms, and builds a model from the perspective of green transformation and development. The research shows that the collaborative development model of new rural production and living civilization construction has a certain effect, and has a certain role in promoting the collaborative development of new rural production and living civilization construction.

## Figures and Tables

**Figure 1:** Wheel selection method.

**Figure 2:** Flowchart of genetic algorithm.

**Figure 3:** Pareto optimal solution in the solution space and Pareto optimal solution in the target space in two-objective planning.

**Figure 4:** Pareto frontier of two-objective optimization.

**Figure 5:** Basic flow chart of multiobjective evolutionary algorithm (MOEA).

**Figure 6:** Schematic diagram of energy flow in the agro-ecosystem.

**Figure 7:** Simulation results for problem 1. (a) The running result of UCEMOA on problem 1. (b) The running results of NSGA-II on problem 1.

**Figure 8:** Simulation results for problem 2. (a) The running result of UCEMOA on problem 2. (b) The running results of NSGA-II on problem 2.

**Figure 9:** Simulation results for problem 3. (a) The running result of UCEMOA on problem 3. (b) The running results of NSGA-II on problem 3.

**Figure 10:** Simulation results for problem 4. (a) The running result of UCEMOA on problem 4. (b) The running results of NSGA-II on problem 4.

**Figure 11:** Evaluation of the effect of the collaborative development model of new rural production and life civilization construction.

**Algorithm 1:** : The algorithm divides the solution space into *H* subspaces.

**Algorithm 2:** : The algorithm generates the initial population.

**Table 1:** The values of *σ*.

Level of each factor	Value for each factor	*σ*
5	2.00-4.00	2.00
7	2.00-6.00	3.00
11	2.00-10.00	7.00

13	2.00	5.00
	3.00	4.00
	4.00-12.00	6.00

17	2.00-16.00	10.00

19	2.00-3.00	8.00
	4.00-18.00	14.00

23	2.00,13.00-14.00, 20.00-22.00	7.00
	8.00-12.00	15.00
	3.00-9.00,1 5.00-19.00	17.00

29	2.00	12.00
	3.00	9.00
	4.00-7.00	16.00
	8.00-12.00, 16.00-34.00	8.00
	13.00-15.	14.00
	25.00-28.00	18.00

31	2.0,5.00-12.00, 20.00-30.00	12.00
	3.00-4.0, 13.00-19.00	22.00

## Data Availability

The labeled datasets used to support the findings of this study are available from the author upon request.

## References

[1] Mdee A., Ofori A., Chasukwa M., Manda S. (2021). Neither sustainable nor inclusive: a political economy of agricultural policy and livelihoods in Malawi, Tanzania and Zambia. *Journal of Peasant Studies*.

[2] Gontard N., Sonesson U., Birkved M. (2018). A research challenge vision regarding management of agricultural waste in a circular bio-based economy. *Critical Reviews in Environmental Science and Technology*.

[3] Sakhno A., Salkova I., Broyaka A., Priamukhina N. (2020). A methodological analysis for the impact assessment of the digitalisation of economy on agricultural growth. *International Journal of Advanced Science and Technology*.

[4] Fortunati S., Morea D., Mosconi E. M. (2020). Circular economy and corporate social responsibility in the agricultural system: cases study of the Italian agri-food industry. *Agricultural Economics*.

[5] Hua J., Wang D. (2018). Research on relationship between agricultural water and agricultural economy based on growth drag of water resources. *Acta Agriculturae Jiangxi*.

[6] Lupenko Y. O., Gutorov A. O., Gutorov O. I. (2018). Investment ensuring for development of integration relations in the agricultural sector of Ukrainian economy. *Financial and credit activity: Problems of Theory and Practice*.

[7] Trukhachev V., Bobrishev A., Khokhlova E., Ivashova V., Fedisko O. (2019). Personnel training for the agricultural sector in terms of digital transformation of the economy: trends, prospects and limitations. *International Journal of Civil Engineering & Technology*.

[8] Radchenko O., Matveyeva M., Holovanova H., Makhyboroda K., Haibura Y. (2020). Information and analytical providion of budget support of institutional sectors of the economy (on the example of the agricultural sector of Ukraine). *Independent Journal of Management & Production*.

[9] Astolfi V., Astolfi A. L., Mazutti M. A. (2019). Cellulolytic enzyme production from agricultural residues for biofuel purpose on circular economy approach. *Bioprocess and Biosystems Engineering*.

[10] Featherstone A. M. (2018). The farm economy: future research and education priorities. *Applied Economic Perspectives and Policy*.

[11] Zharikov R. V., Bezpalov V. V., Lochan S. A., Barashkin M. V., Zharikov A. R. (2018). Economic security of regions as a criterion for formation and development of agricultural clusters by means of innovative technologies. *Scientific Papers Series Management, Economic Engineering in Agriculture and Rural Development*.

[12] Brannstrom C. (2020). Feeding the world: Brazil’s transformation into a modern agricultural economy; agribusiness and the neoliberal food system in Brazil: frontiers and fissures of agro-neoliberalism. *The AAG Review of Books*.

[13] Bergius M., Benjaminsen T. A., Widgren M. (2018). Green economy, Scandinavian investments and agricultural modernization in Tanzania. *Journal of Peasant Studies*.

[14] Ahmed I., Socci C., Severini F., Yasser Q. R., Pretaroli R. (2018). The structures of production, final demand and agricultural output: a Macro Multipliers analysis of the Nigerian economy. *Economia Politica*.

[15] Noviar H., Masbar R., Aliasuddin S. S., Zulham T., Saputra J. (2020). The agricultural commercialisation and its impact on economy management: an application of duality-neoclassic and stochastic frontier approach. *Industrial Engineering & Management Systems*.

[16] Debela M., Diriba S., Bekele H. (2018). Impact of cooperatives membership on economy in eastern oromia: the case of haramaya agricultural FARMERS’COOPERATIVE UNION (hafcu). *Annals of Public and Cooperative Economics*.

[17] Ramsey D., Malcolm C. D. (2018). The importance of location and scale in rural and small town tourism product development: the case of the Canadian Fossil Discovery Centre, Manitoba, Canada. *The Canadian Geographer/Le Géographe canadien*.

[18] Drummond F., Snowball J. (2019). Cultural clusters as a local economic development strategy in rural, small town areas: the sarah baartman district in South Africa. *Bulletin of Geography. Socio-Economic Series*.

[19] Abreu I., Nunes J. M., Mesias F. J. (2019). Can rural development be measured? design and application of a synthetic index to Portuguese municipalities. *Social Indicators Research*.

[20] González Díaz J. A., Celaya R., Fernández García F., Osoro K., Rosa García R. (2019). Dynamics of rural landscapes in marginal areas of northern Spain: past, present, and future. *Land Degradation & Development*.

